# Effect of Danqi Buxin Decoction on Chronic Function Indexes and Life Quality in Patients with Chronic Heart Failure of Yang Deficiency Type

**DOI:** 10.1155/2021/7297361

**Published:** 2021-10-19

**Authors:** Yunjiao Sheng, Hong Qiu, Sijuan Chen

**Affiliations:** ^1^Department of Health Care, Jinan Municipal Hospital of Traditional Chinese Medicine, Jinan 250012, Shandong Province, China; ^2^Central Pharmacy, Qingdao Municipal Hospital, Qingdao 266000, Shandong Province, China; ^3^Cardiology of Department, Jinan Municipal Hospital of Traditional Chinese Medicine, Jinan 250012, Shandong Province, China

## Abstract

**Objective:**

The purpose was to explore the clinical effect of Danqi Buxin decoction on chronic heart failure (CHF) with yang deficiency and its effect on cardiac function and life quality of patients.

**Methods:**

106 CHF patients with yang deficiency treated in Jinan Municipal Hospital of Traditional Chinese Medicine from February 2019 to February 2020 were selected as the research objects and divided into the treatment group and reference group according to the odd and even admission numbers, with 53 cases in each group. The reference group was treated with routine antiheart failure drugs, while the treatment group was additionally treated with Danqi Buxin decoction to compare the clinical effect and cardiac function changes between the two groups.

**Results:**

The clinical effective rate in the treatment group was significantly higher than that in the reference group (*P* < 0.05). The TCM symptom scores at T1, T2, and T3 in the treatment group were significantly higher than those in the reference group (*P* < 0.05). After treatment, the LVEDV levels in both groups were significantly higher than those before treatment, while the BNP levels were significantly lower than those before treatment (*P* < 0.001). The LVEDV level in the treatment group after treatment was higher than that in the reference group, while the BNP level in the treatment group was significantly lower than that in the reference group (*P* < 0.001). The life quality scores in the treatment group after treatment were significantly higher than those in the reference group (*P* < 0.05).

**Conclusion:**

Danqi Buxin decoction on the basis of conventional drugs can significantly improve the cardiac function and life quality of CHF patients with yang deficiency type. Its further research is helpful to establish a good treatment plan for CHF patients.

## 1. Introduction

Chronic heart failure (CHF) is a syndrome in which heart disease develops to the end stage due to various causes. With a high mortality rate, a high hospitalization rate, poor clinical prognosis, and high treatment cost, it brings heavy burden to the family of patients [1, 2]. At present, Western medicine mainly adopts a conservative treatment including angiotensin receptor blockers, *β*-blockers, and other drugs to improve patients' congestion and alleviate the condition. Although significant progress has been made in the treatment of heart failure, there are still many shortcomings, such as side effects caused by vasodilators or diuretics. Besides, long-term administration will lead to lower treatment compliance of patients, failing to achieve the expected therapeutic effect and prolong the survival of patients [3]. Therefore, exploring safe and efficient treatment methods is of great significance to improve the life quality and prolong survival time of patients. Traditional Chinese medicine (TCM) has high safety, and its components and unique combination can play a role of multitarget and comprehensive dialectical treatment [4, 5]. TCM classifies CHF as heart impediment, palpitation edema, and other categories and believes that the disease is a heart qi insufficiency syndrome that occurs mainly in the heart but involves important organs such as the kidney, spleen, and lung [6, 7]. In patients with heart yang deficiency, lack of warm nourishing in blood vessels affects qi-blood circulation and causes qi disorder, resulting in qi stagnation, blood deficiency, and endogenous turbid dampness. Therefore, in the treatment of CHF, especially for patients with heart yang deficiency, the basic principle should be activating blood, dissolving stasis, dredging collaterals, inducing diuresis, and supplementing qi to warm yang [8]. Based on this, to analyze the therapeutic effect of Danqi Buxin decoction on CHF with yang deficiency type, 106 CHF patients with yang deficiency treated in our hospital from February 2019 to February 2020 were selected as the research objects, summarized, and reported as follows.

## 2. Materials and Methods

### 2.1. General Information

106 CHF patients with yang deficiency treated in Jinan Municipal Hospital of Traditional Chinese Medicine from February 2019 to February 2020 were selected as the research objects and divided into the treatment group and reference group according to the odd and even admission numbers, with 53 cases in each group. The treatment group had 29 males and 24 females, with an average age of (54.38 ± 3.49) years old and an average disease course of (3.08 ± 0.32) years. The number of cases with cardiac functions II, III, and IV was 8, 34, and 11, while the average Lee's score of heart failure was (13.46 ± 1.27). The reference group had 28 males and 25 females, with an average age of (54.42 ± 3.45) years old and an average disease course of (3.11 ± 0.26) years. The number of cases with cardiac functions II, III, and IV was 6, 37, and 10, while the average Lee's score of heart failure was (13.53 ± 1.32). There was no significant difference in the baseline data between the two groups (*P* < 0.05) indicating comparability. The flow diagram is shown in Figure 1.

### 2.2. Inclusion Criteria

① The patients met the diagnostic criteria of CHF in Guidelines for Diagnosis and Treatment of Chronic Heart Failure [9], with the clinical manifestations such as edema of both lower limbs, exertional dyspnea, and fatigue; ② the patient met the TCM diagnostic criteria of yang deficiency type in Guidelines for the Clinical Research of Chinese Medicine New Drugs [10], including fatigue, shortness of breath, and edema, with subsymptoms such as abdominal distension, cold body, and cold limbs; ③ the cardiac function of the patients were grades II–IV according to New York Heart Association (NYHA) classification of cardiac function; and ④ this study was approved by the Ethics Committee of Jinan Municipal Hospital of Traditional Chinese Medicine, and all patients had signed the informed consent.

### 2.3. Exclusion Criteria

① The patients had severe liver and kidney dysfunction; ② the patients were complicated with malignant arrhythmia or acute myocardial infarction; ③ the patients were allergic to Danqi Buxin decoction and other drug ingredients used in this study; and ④ the patients were complicated with malignant tumors.

## 3. Methods

Both groups of patients were given basic treatment (diuretic, oxygen inhalation, cardiotonic, and antiinfection treatment), limiting the intake of water and sodium, paying attention to rest, correcting arrhythmia, and maintaining electrolyte and acid-base balance. The reference group was treated with routine antiheart failure drugs, including 20 mg of oral spironolactone (SFDA approval no.: H33020070; manufacturer: Hangzhou Minsheng Pharmaceutical Co., Ltd.; specification: 20 mg*∗*100 s), 0.125 mg of digoxin (SFDA approval no.: H37020332; manufacturer: Shandong Xinhua Pharmaceutical Co., Ltd.; specification: 0.25 mg), and 0.5 mg of nitroglycerin (SFDA approval no.: H13022503; manufacturer: Hebei Medical University Pharmaceutical Factory; specification: 0.5 mg × 100 tablets/bottle). The above three drugs were taken once daily. On this basis, the treatment group was additionally treated with Danqi Buxin decoction with the formula including 15 g of Bighead Atractylodes Rhizome, 15 g of dried tangerine peel, 15 g of root of red-rooted *Salvia*, 15 g of Chinese angelica, 15 g of Rhizoma Chuanxiong, 15 g of Cassia Twig, 10 g of sun-dried ginseng, 10 g of dwarf lilyturf tuber, and 30 g of *Astragalus mongholicus*, one dose each day. Cooked in water to obtain 150 ml of juice, the decoction was warmly taken three times a day, with 50 ml each time. Both groups of patients were continuously treated for 14 days.

### 3.1. Evaluation Indexes

Clinical efficacy evaluation: relevant criteria in Guidelines for the Clinical Research of Chinese Medicine New Drugs were used to evaluate the clinical efficacy. After treatment, all clinical symptoms disappeared, and NYHA classification reached grade I, which was cured; The symptoms were significantly improved, and NYHA classification reached grade I or increased by 2 grades, which was markedly effective. The symptoms were improved, and NYHA classification increased by 1 grade, which was effective. The symptoms and NYHA classification were not improved, or the condition was aggravated, which was ineffective. Treatment effective rate = cured rate + markedly effective rate + effective rate.

According to TCM scores corresponding to the degree of clinical symptoms, the TCM symptom scores of patients before treatment (T0), 5 days after treatment (T1), 10 days after treatment (T2), and 14 days after treatment (T3) were calculated and compared between the two groups.

Echocardiography was used to detect the left ventricular end-diastolic volume (LVEDV) levels of both groups before and after treatment. 5 ml of fasting venous blood was collected from the two groups before and after treatment. After anticoagulation with heparin sodium and centrifugation, the serum was extracted for detection. BNP-Triage kits (manufacturer: Shanghai Westang Biotech Co., Ltd.) were used to determine the BNP level.

The daily quality of life scale for patients with chronic heart failure made by our department was used to evaluate the life quality of both groups after treatment, including disease condition, physical strength, living function, social psychological function, and working condition. The total score was 30 points in condition and social psychological function, 100 points in physical strength, 20 points in living function, and 15 points in working condition. A higher score indicated higher life quality of patients.

### 3.2. Statistical Methods

All the experimental data were statistically analyzed and processed by SPSS 21.0 software, and the data were graphed by GraphPad Prism 7 (GraphPad Software, San Diego, USA). The count data were tested by *X*^2^, expressed by (*n* (%)), and the measurement data were measured by the *t*-test, expressed by $\left(\bar{x}\pm s\right)$. The difference was statistically significant when *P* < 0.05.

## 4. Results

### 4.1. Comparison of Demographic Characteristics between the Two Groups

No notable differences in demographic characteristics were observed between the two groups (*P* < 0.05; Table 1).

### 4.2. Comparison of Clinical Efficacy between the Two Groups

The total clinical effective rate in the treatment group was significantly higher than that in the reference group (*P* < 0.05, Table 2).

### 4.3. Comparison of TCM Symptom Scores at Different Time between the Two Groups

The TCM symptom scores at T1, T2, and T3 in the treatment group were significantly higher than those in the reference group (*P* < 0.05, Figure 2).

### 4.4. Comparison of LVEDV and BNP Levels before and after Treatment between the Two Groups

After treatment, the LVEDV levels in both groups were significantly higher than those before treatment, while the BNP levels were significantly lower than those before treatment (*P* < 0.001, Figures 2 and 3). The LVEDV level in the treatment group after treatment was higher than that in the reference group, while the BNP level was significantly lower than that in the reference group (*P* < 0.001, Figures 3 and 4).

### 4.5. Comparison of Life Quality Scores after Treatment between the Two Groups

After treatment, the scores of disease condition, physical strength, living function, social psychological function, and working condition in the treatment group were significantly higher than those in the reference group (*P* < 0.05, Table 3).

## 5. Discussion

Clinical investigation shows that CHF is a chronic progressive disease, and about 25% of patients have the risk of secondary hospitalization, which seriously affects their life quality. Since decreased myocardial contractility and cardiac hemodynamic overload are the main causes of CHF, the basic treatment principle in clinics is to rebuild myocardial cells and restore cardiac function [11]. TCM has accumulated a lot of experience in the treatment of cardiovascular diseases and believes that heart yang deficiency is the root of heart failure. Heart failure has gradually evolved from heart qi insufficiency to heart yang deficiency, which is caused by the weakness of heart qi and yang, and runs through the whole process of disease occurrence and development [12]. Although Western medicine has made significant progress in CHF treatment, there are still many shortcomings, such as the side effects of drugs which lead to malignant arrhythmia, affecting the therapeutic effect [13, 14]. TCM believes that attention should be paid to yin-yang balance and the recovery of various organ functions in treatment, thus improving clinical symptoms and life quality.

TCM believes that CHF is mostly due to damage of viscera caused by congenital deficiency or acquired pathogenic factors [15]. In this study, the CHF patients with yang deficiency were treated with Danqi Buxin decoction on the basis of routine antiheart failure drugs. After treatment, the LVEDV levels in both groups were significantly higher than those before treatment (*P* < 0.001), and the LVEDV level in the treatment group was significantly higher than that in the reference group (*P* < 0.001). In Danqi Buxin decoction, root of red-rooted *Salvia* cools blood, eliminates carbuncle, improves blood circulation, and disperses stasis; dwarf lilyturf tuber tonifies the stomach, promotes fluid, and nourishes yin to moisten the lung; sun-dried ginseng has the effect of invigorating primordial energy, nourishing blood, and tranquilizing mind by nourishing the heart. Therefore, it is speculated that the whole prescription has the effect of reducing myocardial oxygen consumption and improving coronary blood flow, which effectively reduces the clinical symptoms and improves prognosis of CHF patients [16]. Moreno-Suarez et al. [17] pointed out in their study that after CHF patients were treated with Shenqi Fumai decoction based on the routine Western medicine treatment, the LVEDV level after treatment was significantly higher than that before treatment, indicating that TCM decoction can activate blood, remove stasis, dredge collaterals, induce diuresis, and supplement qi to warm yang, thereby improving the cardiac function and clinical symptoms of CHF patients. Improving the quality of life of CHF patients is not only one of the goals of clinical treatment but also an important indicator to measure the therapeutic effect of heart failure. This study evaluated the effect of different treatment regimens on the quality of life of CHF patients by using self-made quality of life scale, and the results showed that the scores in the treatment group after treatment were notably higher compared with the reference group (*P* < 0.001). It is possibly because Danqi Buxin decoction has the effects of warming yang, invigorating qi, and inducing diuresis to alleviate edema, thereby alleviating clinical symptoms and improving the life quality of patients. The study includes the following deficiencies. (1) This study is a clinical trial including 106 cases and 2 weeks of treatment, with short observation cycle, small sample size, and patients all coming from our hospital. Therefore, it is necessary to carry out more multicenter studies with a larger sample size and longer follow-up. (2) This study only includes preliminary observation on the curative effect and lacks the research on the readmission rate and the long-term quality of life, which needs further clinical verification.

In conclusion, Danqi Buxin decoction can significantly improve the cardiac function and life quality of CHF patients with yang deficiency type, with a significant effect, which is worthy of clinical promotion and application.

## Figures and Tables

**Figure 1:** Flow diagram of the study.

**Figure 2:** Comparison of TCM symptom scores at different time between the two groups $\left(\bar{x}\pm s\right)$. Note: the abscissa represents T0, T1, T2, and T3, and the ordinate represents the TCM symptom score (points). The TCM symptom scores of the treatment group at T0, T1, T2, and T3 were (13.69 ± 0.74), (9.05 ± 0.34), (7.92 ± 0.17), and (6.35 ± 0.14), respectively. The TCM symptom scores of the reference group at T0, T1, T2, and T3 were (13.64 ± 0.71), (11.32 ± 0.29), (9.63 ± 0.23), and (8.07 ± 0.25), respectively. ^*∗*^Significant difference in the TCM symptom scores at T1 between the two groups (*t* = 36.981, *P* < 0.001). ^*∗∗*^Significant difference in the TCM symptom scores at T2 between the two groups (*t* = 45.527, *P* < 0.001). ^*∗∗∗*^Significant difference in the TCM symptom scores at T3 between the two groups (*t* = 43.701, *P* < 0.001).

**Figure 3:** Comparison of LVEDV levels before and after treatment between the two groups $\left(\bar{x}\pm s\right)$. Note: the abscissa represents before treatment and after treatment, and the ordinate represents the LVEDV level (ml). The LVEDV levels of the treatment group before and after treatment were (0.41 ± 0.06) ml and (0.63 ± 0.09) ml, respectively. The LVEDV levels of the reference group before and after treatment were (0.42 ± 0.04) ml and (0.51 ± 0.11) ml, respectively. ^*∗*^Significant difference in the LVEDV levels of the treatment group before and after treatment (*t* = 14.807, *P* < 0.001). ^*∗∗*^Significant difference in the LVEDV levels of the reference group before and after treatment (*t* = 5.598, *P* < 0.001). ^*∗∗∗*^Significant difference in the LVEDV levels between the two groups after treatment (*t* = 6.147, *P* < 0.001).

**Figure 4:** Comparison of BNP levels before and after treatment between the two groups $\left(\bar{x}\pm s\right)$. Note: the abscissa represents before treatment and after treatment, and the ordinate represents the BNP level (pg/ml). The BNP levels of the treatment group before and after treatment were (175.34 ± 13.78) pg/ml and (91.44 ± 10.33) pg/ml, respectively. The BNP levels of the reference group before and after treatment were (175.41 ± 13.69) pg/ml and (115.48 ± 11.62) pg/ml, respectively. ^*∗*^Significant difference in the BNP levels of the treatment group before and after treatment (*t* = 34.466, *P* < 0.001). ^*∗∗*^Significant difference in the BNP levels of the reference group before and after treatment (*t* = 24.297, *P* < 0.001). ^*∗∗∗*^Significant difference in the BNP levels between the two groups after treatment (*t* = 11.257, *P* < 0.001).

**Table 1:** Comparison of demographic characteristics between the two groups.

Items	Treatment group	Reference group	*X* ^2^/*t*	*P*
Education level				
Primary school	10 (18.87)	11 (20.75)	0.059	0.807
Junior high school	27 (50.94)	30 (56.60)	0.342	0.559
Senior high school	11 (20.75)	9 (16.98)	0.247	0.620
University and above	5 (9.43)	3 (5.66)	0.541	0.462
Occupation				
Peasant	23 (43.40)	26 (49.06)	0.342	0.559
Worker	18 (33.96)	15 (28.30)	0.396	0.529
Teacher	8 (15.09)	5 (9.43)	0.789	0.374
Others	4 (7.55)	7 (13.21)	0.913	0.339
Residence			0.604	0.437
Urban area	25 (47.17)	29 (54.72)		
Rural area	28 (52.83)	24 (45.28)		
Marital status				
Married	49 (92.45)	47 (88.68)	0.442	0.506
Unmarried	2 (3.77)	1 (1.89)	0.343	0.558
Divorced	2 (3.77)	5 (9.43)	1.377	0.241

**Table 2:** Comparison of clinical efficacy between the two groups (*n* (%)).

Group	*n*	Cured	Markedly effective	Effective	Ineffective	Total effective rate
Treatment group	53	23 (43.40%)	25 (47.17%)	2 (3.77%)	3 (5.66%)	90.57% (48/53)
Reference group	53	15 (28.30%)	20 (37.74%)	8 (15.09%)	10 (18.87%)	66.04% (35/53)
*X* ^2^						4.296
*P*						<0.05

**Table 3:** Comparison of life quality scores after treatment between the two groups ($\bar{x}\pm s$, points).

Group	*n*	Disease condition	Physical strength	Living function	Social psychological function	Working condition
Treatment group	53	21.43 ± 1.18	57.82 ± 2.76	15.22 ± 2.26	23.68 ± 1.98	7.61 ± 0.69
Reference group	53	16.52 ± 1.23	50.47 ± 2.33	10.49 ± 2.17	16.92 ± 1.65	4.62 ± 0.52
*t*		20.971	14.814	10.991	19.094	25.194
*P*		<0.001	<0.001	<0.001	<0.001	<0.001

## Data Availability

The data used to support the findings of this study are available from the corresponding author upon request.
